RETRACTED

# Identification of a Novel Gammaretrovirus in Prostate Tumors of Patients Homozygous for R462Q *RNASEL* Variant

**DOI:** 10.1371/journal.ppat.0020025

**Published:** 2006-03-31

**Authors:** Anatoly Urisman, Ross J Molinaro, Nicole Fischer, Sarah J Plummer, Graham Casey, Eric A Klein, Krishnamurthy Malathi, Cristina Magi-Galluzzi, Raymond R Tubbs, Don Ganem, Robert H Silverman, Joseph L DeRisi

**Affiliations:** 1 Department of Biochemistry and Biophysics, University of California San Francisco, San Francisco, California, United States of America; 2 Department of Cancer Biology, Lerner Research Institute, Cleveland Clinic, Cleveland, Ohio, United States of America; 3 Department of Chemistry, Cleveland State University, Cleveland, Ohio, United States of America; 4 Department of Microbiology and Immunology, University of California San Francisco, San Francisco, California, United States of America; 5 Glickman Urological Institute, Cleveland Clinic, Cleveland, Ohio, United States of America; 6 Anatomic and Clinical Pathology, Cleveland Clinic, Cleveland, Ohio, United States of America; 7 Department of Medicine, University of California San Francisco, San Francisco, California, United States of America; 8 Howard Hughes Medical Institute, University of California San Francisco, San Francisco, California, United States of America; University of Pennsylvania School of Medicine, United States of America

## Abstract

Ribonuclease L (RNase L) is an important effector of the innate antiviral response. Mutations or variants that impair function of RNase L, particularly R462Q, have been proposed as susceptibility factors for prostate cancer. Given the role of this gene in viral defense, we sought to explore the possibility that a viral infection might contribute to prostate cancer in individuals harboring the R462Q variant. A viral detection DNA microarray composed of oligonucleotides corresponding to the most conserved sequences of all known viruses identified the presence of gammaretroviral sequences in cDNA samples from seven of 11 R462Q-homozygous (QQ) cases, and in one of eight heterozygous (RQ) and homozygous wild-type (RR) cases. An expanded survey of 86 tumors by specific RT-PCR detected the virus in eight of 20 QQ cases (40%), compared with only one sample (1.5%) among 66 RQ and RR cases. The full-length viral genome was cloned and sequenced independently from three positive QQ cases. The virus, named XMRV, is closely related to xenotropic murine leukemia viruses (MuLVs), but its sequence is clearly distinct from all known members of this group. Comparison of *gag* and *pol* sequences from different tumor isolates suggested infection with the same virus in all cases, yet sequence variation was consistent with the infections being independently acquired. Analysis of prostate tissues from XMRV-positive cases by in situ hybridization and immunohistochemistry showed that XMRV nucleic acid and protein can be detected in about 1% of stromal cells, predominantly fibroblasts and hematopoietic elements in regions adjacent to the carcinoma. These data provide to our knowledge the first demonstration that xenotropic MuLV-related viruses can produce an authentic human infection, and strongly implicate RNase L activity in the prevention or clearance of infection in vivo. These findings also raise questions about the possible relationship between exogenous infection and cancer development in genetically susceptible individuals.

RETRACTED

## Synopsis

Prostate cancer is the most frequent cancer and the second leading cause of cancer deaths in US men over the age of 50. Several genetic factors have been proposed as potential risk factors for the development of prostate cancer, including a viral defense gene called *RNASEL*. A common genetic variant in this gene, R462Q, was recently implicated in up to 13% of prostate cancer cases. Given the antiviral role of *RNASEL,* the authors sought to examine if a virus might be present in prostate cancers associated with the R462Q variant. Using a DNA microarray designed to detect all known viral families, the authors identified a novel virus, named XMRV, in a subset of prostate tumor samples. Polymerase chain reaction testing of 86 prostate tumors for the presence of XMRV revealed a strong association between the presence of the virus and being homozygous for the R462Q variant. Cloning and sequencing of the virus showed that XMRV is a close relative of several known xenotropic murine leukemia viruses. This report presents the first documented cases of human infection with a xenotropic retrovirus. Future work will address the potential connection between XMRV infection and the increased prostate cancer risk in patients with the R462Q *RNASEL* variant.

## Introduction

Type I interferons (IFNs) are rapidly mobilized in response to viral infection and trigger potent antiviral responses. One such response is the induction by IFN of a family of 2′5′ oligoadenylate synthetases (OAS); upon activation by virally encoded dsRNA, these enzymes produce 5′-phosphorylated 2′-5′ linked oligoadenylates (2–5A) from ATP [1]. 2–5A, in turn, is an activator of ribonuclease L (RNase L) [2], which degrades viral (and cellular) single stranded RNAs [3]. In vivo evidence for the antiviral role of the 2–5A system was provided by studies with RNase L^−/−^ mice, which have enhanced susceptibility to infections by the picornaviruses, encephalomyocarditis virus, and Coxsackievirus B4 [4,5]. Ultimately, sustained activation of RNase L triggers a mitochondrial pathway of apoptosis that eliminates virus-infected cells [4,6–8]. Genetic lesions in RNase L impair this apoptotic response, which has raised interest in the possibility that such mutations might also contribute to malignancy [9].

RETRACTED

In this context, several recent studies have linked germline mutations in RNase L to prostate cancer susceptibility [10–13]. Prostate cancer has a complex etiology influenced by androgens, diet, and other environmental and genetic factors [14]. While sporadic prostate cancer displays an age-related increase in prevalence, familial prostate cancer kindreds often display early-onset disease. Such kindreds, defined by having more than three affected members per family, account for 43% of early onset cases (<55 years old) and 9% of all cases [15]. The genetics of hereditary prostate cancer (HPC) is complex, and several genes have been proposed as susceptibility factors in this syndrome. Interestingly, one of these, *HPC1,* is linked to *RNASEL* [10,11]. Several germline mutations or variants in *HPC1/RNASEL* have been observed in HPC [10–13] (reviewed in [16]), including a common (35% allelic frequency) missense variant of RNase L, in which a G to A transition at nucleotide (nt) position 1385 (G1385A) results in a glutamine instead of arginine at amino acid position 462 (R462Q). Remarkably, a large, controlled sib-pair study implicated the R462Q RNase L variant in up to 13% of unselected prostate cancer cases [11]. One copy of the mutated gene increased the risk of prostate cancer by about 50%, whereas individuals that were homozygous for the mutation had a 2-fold increased risk of prostate cancer. The R462Q RNase L variant had a 3-fold decrease in catalytic activity compared with the wild-type enzyme [9,11]. However, while several case-controlled genetic and epidemiologic studies support the involvement of *RNASEL* (and notably the R462Q variant) in prostate cancer etiology [10–13], others do not [17–19], suggesting that either population differences or environmental factors may modulate the impact of *RNASEL* on prostatic carcinogenesis.

While the antiapoptotic phenotype of RNase L deficiency has dominated previous discussions of its possible linkage to cancer, RNase L is also a key effector of the antiviral action of interferons. This led us to consider the possibility that the putative linkage of RNase L alterations to HPC might reflect enhanced susceptibility to a viral agent. To test this hypothesis, we have examined RNA derived from wild-type and RNase L variant (R462Q) prostate tumors for evidence of viral sequences, by hybridization to a DNA microarray composed of the most conserved sequences of all known human, animal, plant, and bacterial viruses [20,21]. Here we report that 40% (eight of 20) of all tumors homozygous for the R462Q allele harbored the genome of a distinct gammaretrovirus closely related to xenotropic murine leukemia viruses (MuLVs). In contrast, retroviral sequences were present in <2% of tumors bearing at least one copy of the wild-type allele (one of 66). In addition, virus-harboring cells were detected within infected prostatic tumor tissues by fluorescence in situ hybridization (FISH) and immunohistochemistry (IHC). These findings represent the first detection of xenotropic MuLV–like agents in humans, and reveal a strong association between infection with the virus and defects in RNase L activity. The relation of retroviral infection to prostate cancer will require further study, but a cofactor role is not excluded.

RETRACTED

## Results

### Detection of XMRV by Microarray-Based Screening

To search for potential viruses in prostate cancer tumors, we employed a DNA microarray-based strategy designed to screen for viruses from all known viral families [20,21]. Total or polyadenylated RNA extracted from tumor tissue was first amplified and fluorescently labeled in a sequence-nonspecific fashion. The amplified and labeled fragments, which contained host as well as potential viral sequences, were then hybridized to a DNA microarray (Virochip, University of California San Francisco, San Francisco, United States) bearing the most conserved sequences of ~950 fully sequenced NCBI reference viral genomes (~11,000 70-mer oligonucleotides).

The Virochip was used to screen RNA samples isolated from prostate tumors of 19 individuals (Figure 1). A positive hybridization signal suggestive of a gammaretrovirus was detected in seven of 11 tumors from patients homozygous for the R462Q *RNASEL* variant (QQ). In contrast, no virus was detected in three tumors from RQ heterozygotes, and only one of five tumors from RR individuals was positive. Clustering of the microarray oligonucleotide intensities (Figure 1) revealed a similar hybridization pattern in all positive cases. Furthermore, a computational analysis using E-Predict, a recently described algorithm for viral species identification [22], suggested that the same or similar mammalian gammaretrovirus was present in all positive tumors (Table S1). Thus, the Virochip detected the presence of a probable gammaretrovirus in half of the QQ tumor samples and in only one non-QQ sample.

**Figure 1:** XMRV Detection by DNA Microarrays and RT-PCR (A) Virochip hybridization patterns obtained for tumor samples from 19 patients. The samples (*x-*axis) and the 502 retroviral oligonucleotides present on the microarray (*y-*axis) were clustered using hierarchical clustering. The red color saturation indicates the magnitude of hybridization intensity. (B) Magnified view of a selected cluster containing oligonucleotides with the strongest positive signal. Samples from patients with QQ *RNASEL* genotype are shown in red, and those from RQ and RR individuals as well as controls are in black. (C) Results of nested RT-PCR specific for XMRV *gag* gene. Amplified *gag* PCR fragments along with the corresponding human *GAPDH* amplification controls were separated by gel electrophoresis using the same lane order as in the microarray cluster.

RETRACTED

### Characterization of XMRV Genome

To further characterize the virus, we recovered its entire genome from one of the tumors (VP35) (Figure 2). To obtain viral clones, we first employed a direct microarray recovery technique described previously [21]. Briefly, amplified nucleic acid from the tumor tissue, which hybridized to viral microarray oligonucleotides, was eluted from two specific spots. The eluted DNA was re-amplified, and plasmid libraries constructed from this material were screened by colony hybridization using the spots' oligonucleotides as probes. The array oligonucleotides used in this case derived from the LTR region of murine type C retrovirus (MTCR) and spleen focus-forming virus (SFFV) [23]. The largest recovered fragment was 415 nt in length, and had 96% nt identity to the LTR region of MTCR, a MuLV identified in the genome of a mouse myeloma cell line (T. Heinemeyer, unpublished data). These findings established that the virus in question was indeed a gammaretrovirus, and likely a relative of MuLVs. To clone and sequence the rest of the viral genome from sample VP35, we used tumor cDNA to PCR-amplify overlapping segments using primers derived from MTCR; gaps were closed using primers from earlier recovered clones (Figure 2B and Table S2). Using a similar strategy, we have also determined the full sequence of the virus from a second tumor, VP42. Finally, a complete viral genomic sequence from a third tumor case, VP62, was obtained by PCR amplification of two ~4 Kb–long overlapping fragments jointly spanning close to the entire length of the virus (Figure 2B). The three sequenced genomes share >98% nt identity overall and >99% amino acid (aa) identity for predicted open reading frames (ORFs), and thus represent the same virus.

**Figure 2:** Complete Genome of XMRV (A) Schematic map of the 8185 nt XMRV genome. LTR regions (R, U5, U3) are indicated with boxes. Predicted open reading frames encoding Gag, Gag-Pro-Pol, and Env polyproteins are labeled in green. The corresponding start and stop codons (AUG, UAG, UGA, UAA) as well as the alternative Gag start codon (CUG) are shown with their nt positions. Similarly, splice donor (SD) and acceptor (SA) sites are shown and correspond to the spliced 3.2-Kb Env subgenomic RNA (wiggled line). (B) Cloning and sequencing of XMRV VP35 and VP62 genomes. Clones obtained by probe recovery from hybridizing microarray oligonucleotides (blue bar) or by PCR from tumor cDNA (black bars) were sequenced. Primers used to amplify individual clones (Table S2) were derived either from the genome of MTCR (black arrows) or from overlapping VP35 clones (blue arrows). (C) Genome sequence similarity plots comparing XMRV VP35 with XMRV VP42, XMRV VP62, MuLV DG-75, MTCR, and a set of representative non-ecotropic proviruses (mERVs) (see Materials and Methods). The alignments were made using AVID [81], and plots were generated using mVISTA [82] with the default window size of 100 nt. *Y*-axis scale for each plot represents percent nt identities from 50% to 100%. Sequences are labeled as xenotropic (X), polytropic (P), or modified polytropic (Pm).

RETRACTED

The full genome of the virus (Figures 2 and S1) is 8,185 nt long and is distinct from all known isolates of MuLV. The genome is most similar to the genomes of exogenous MuLVs, DG-75 cloned from a human B-lymphoblastoid cell line [24], and MTCR, with which it shares 94% and 93% overall nt sequence identity, respectively. The genome also shares up to 95% nt identity with several full-length Mus musculus endogenous proviruses (Figure 2C). Phylogenetic trees constructed using available mammalian type C retroviral genomes and representative full-length proviral sequences from the mouse genome (Figures 3 and S2) showed that the newly identified virus is more similar to xenotropic and polytropic than to ecotropic genomes. Based on these findings we propose the provisional name Xenotropic MuLV-related virus (XMRV) for this agent.

**Figure 3:** Phylogenetic Analysis of XMRV Based on Complete Genome Sequences Complete genomes of XMRV VP35, VP42, and VP62 (red); MTCR; MuLVs DG-75, AKV, Moloney, Friend, and Rauscher; feline leukemia virus (FLV); koala retrovirus (KoRV); gibbon ape leukemia virus (GALV); and a set of representative non-ecotropic proviruses (mERVs) were aligned using ClustalX (see Materials and Methods). An unrooted neighbor-joining tree was generated based on this alignment, excluding gaps and using Kimura's correction for multiple base substitutions. Bootstrap values (*n* = 1000 trials) are indicated as percentages. Sequences are labeled as xenotropic (X), polytropic (P), modified polytropic (Pm), or ecotropic (E).

RETRACTED

Translation of the XMRV genomic sequence using ORF Finder [25] identified two overlapping ORFs coding for the full-length Gag-Pro-Pol and Env polyproteins. No exogenous coding sequences, such as viral oncogenes, could be detected in the XMRV genome. The predicted Gag polyprotein is 536 aa long and is most similar to a xenotropic provirus on M. musculus Chromosome 9, with which it shares 97% aa identity (Figure S2A). The Pro-Pol polyprotein is 1,197 aa long and has the highest aa identity with MuLV DG-75 and a xenotropic provirus on M. musculus Chromosome 4, 97% and 96%, respectively (Figure S2B). An amber (UAG) stop codon separates the Gag and Pro-Pol coding sequences, analogous to other MuLVs in which a translational read-through is required to generate the full-length Gag-Pro-Pol polyprotein (reviewed in [26]).

Similar to other MuLVs [23,24,27–31], the Env polyprotein of XMRV is in a different reading frame compared with Gag-Pro-Pol. The Env protein sequence is 645 aa long, and has the highest amino acid identity with the Env protein of an infectious MuLV isolated from a human small cell lung cancer line NCI-417 [32] and MuLV New Zealand Black 9–1 xenotropic retrovirus (NZB-9–1) [28]), 95% and 94%, respectively. The XMRV Env protein also shares similarly high identity with several murine xenotropic proviruses (Figure S2C). Conserved splice donor (AGGTAAG, position 204) and acceptor (CACTTACAG, position 5,479) sites involved in the generation of *env* subgenomic RNAs [33] were found in the same relative locations as in other MuLV genomes. A multiple sequence alignment of XMRV Env and corresponding protein sequences of other representative MuLVs (Figure 4) showed that within three highly variable regions (VR), VRA, VRB, and VRC, known to be important for cellular tropism [34–36], XMRV has the highest aa identity with xenotropic envelopes from MuLVs NZB-9–1, NFS-Th-1 [37], and DG-75. Although unique-to-XMRV aa are present in each of the three VRs, based on the overall similarity to the known xenotropic envelopes, we predict that the cellular receptor for XMRV is XPR1 (SYG1), the recently identified receptor for xenotropic and polytropic MuLVs [38–40].

**Figure 4:** Multiple-Sequence Alignment of Protein Sequences from XMRV and Related MuLVs Spanning SU Glycoprotein VRA, VRB, and VRC, Known to Determine Receptor Specificity Env protein sequence from XMRV (identical in VP35, VP42, and VP62; red); MTCR; MuLVs DG-75, NZB-9–1, NFS-Th-1, MCF247, AKV, Moloney, Friend, and Rauscher; and polytropic proviruses MX27 and MX33 [77] were aligned using ClustalX. Sequences are labeled as xenotropic (X), polytropic (P), modified polytropic (Pm), or ecotropic (E). VRs are boxed. Dots denote residues identical to those from XMRV, and deleted residues appear as spaces.

RETRACTED

The long terminal repeat (LTR) of XMRV is 535 nt long and has the highest nt identity with the LTRs from xenotropic MuLVs NFS-Th-1 (96%) and NZB-9–1 (94%). The XMRV LTRs contain known structural and regulatory elements typical of other MuLV LTRs [33,41]. In particular, the CCAAT box, TATAAAA box, and AATAAA polyadenylation signal sequences were found in U3 at their expected locations (Figure S3A). U3 also contains a glucocorticoid response element sequence AGA ACA GAT GGT CCT. Essentially identical sequences are present in genomes of other MuLVs. These elements have been shown to activate LTR-directed transcription and viral replication in vitro in response to various steroids including androgens [42–45]. In addition, presence of an intact glucocorticoid response element is thought to be the determinant of higher susceptibility to FIS-2 MuLV infection in male compared with female NMRI mice [46,47]. Despite these similarities, single nt substitutions unique to XMRV and an insertion of an AG dinucleotide immediately downstream from the TATA box are present in U3 (Figure S3A). Consistent with these findings, a phylogenetic analysis based on U3 sequences from XMRV and from representative xenotropic MuLV provirus groups [48,49] showed that XMRV U3 sequences formed a well-separated cluster most similar to the group containing NFS-Th-1 and NZB-9–1 (Figure S3B).

The 5′ *gag* leader of XMRV, defined as the sequence extending from the end of U5 to the ATG start codon of *gag,* consists of a conserved non-coding region of ~200 nt, containing a proline tRNA primer binding site as well as sequences required for viral packaging [50,51] and the initiation of translation [52,53]. The non-coding region is followed by a ~270-nt region extending from the conserved CTG alternative start codon of *gag.* This region represents the most divergent segment of the genome compared with other MuLVs (Figures 5 and 2C). Unlike ecotropic MuLVs, where translation from this codon adds an ~90 aa N-terminal leader peptide in frame with the rest of the Gag protein, thus generating a glycosylated form of Gag [54], XMRV has a stop codon 53 aa residues downstream from the alternative start. Interestingly, both MuLV DG-75 and MTCR *gag* leader sequences are also interrupted by stop codons, and therefore are not expected to produce full-length glyco-Gag. Furthermore, a characteristic 24-nt deletion was present in this region of the XMRV genome, which is not found in any known exogenous MuLV isolate. However, a shorter deletion of nine nt internal to this region is present in the sequences of several non-ecotropic MuLV proviruses found in the sequenced mouse genome (Figure 5). In cell culture, expression of intact glyco-Gag is not essential for viral replication [55,56]. However, lesions in this region have been associated with interesting variations in pathogenetic properties in vivo [57–61]. For example, an alteration in ten nt affecting five residues in the N-terminal peptide of glyco-Gag was found to be responsible for a 100-fold difference in the frequency of neuroinvasion observed between CasFrKP and CasFrKP41 MuLV strains [62]. In addition, insertion of an octanucleotide resulting in a stop codon downstream of the CUG start codon prevented severe early hemolytic anemia and prolonged latency of erythroleukemia in mice infected with Friend MuLV [58]. While we do not yet know the pathogenetic significance of the lesions in XMRV glyco-Gag, the high degree of sequence divergence suggests that this region may be under positive selective pressure and therefore may be relevant to the establishment of infection within the human host.

RETRACTED

**Figure 5:** Multiple-Sequence Alignment of 5′ *gag* Leader Nucleotide Sequences from XMRV and Related MuLVs Sequences extending from the alternative CUG start codon to the AUG start codon (underlined) of *gag* derived from XMRV VP35, VP42, and VP62 (blue); MTCR, MuLVs DG-75, and Friend; and a set of representative non-ecotropic proviruses (mERVs) were aligned with ClustalX (see Materials and Methods). Predicted amino acid translation corresponding to the VP35 sequence is shown above the alignment (red); asterisk indicates a stop. Sequences are labeled as xenotropic (X), polytropic (P), modified polytropic (Pm), or ecotropic (E). Dots denote nt identical to those from XMRV, and deleted nt appear as spaces.

### Association of XMRV Infection and R462Q *RNASEL* Genotype

To further examine the association between presence of the virus and the R462Q (1385G->A) *RNASEL* genotype, we developed a specific nested RT-PCR assay based on the virus sequence recovered from one of the tumor samples (VP35, see above). The primers in this assay (Figure S1) amplify a 380-nt fragment from the divergent 5′ leader and the N-terminal end of *gag*. The RT-PCR was positive in eight (40%) of 20 examined tumors from homozygous (QQ) individuals. In addition, one tumor from a homozygous wild-type (RR) patient was positive among 52 RR and 14 RQ tumors examined (Figure 1 and Table 1). Interestingly, this case was associated with the highest tumor grade among all XMRV-positive cases (Table S3). PCR specific for the mouse *GAPDH* gene was negative in all samples (unpublished data), arguing strongly against the possibility that the tumor samples were contaminated with mouse nucleic acid. Collectively, these data demonstrate a strong association between the homozygous (QQ) R462Q *RNASEL* genotype and presence of the virus in the tumor tissue (*p* < 0.00002 by two-tail Fisher's exact test).

RETRACTED

**Table 1:** XMRV Screening by *gag* Nested RT-PCR

### XMRV Sequence Diversity in Samples from Different Patients

To examine the degree of XMRV sequence diversity in different patients, we sequenced the amplified fragments from all nine samples, which were positive by the nested *gag* RT-PCR. The amplified *gag* fragments were highly similar (Figure 6A) with >98% nt and >98% aa identity to each other. In contrast, the fragments had <89% nt and <95% aa identity with the most related exogenous sequence of MuLV DG-75. Several corresponding endogenous non-ecotropic sequences were more similar to the XMRV fragments, including the xenotropic provirus from M. musculus Chromosome 9, which was <98% identical on the nt level. Nevertheless, all XMRV-derived fragments were more similar to each other than they were to any other sequence.

**Figure 6:** Comparison of XMRV Sequences Derived from Tumor Samples of Different Patients (A) Phylogenetic tree based on the 380 nt XMRV *gag* RT-PCR fragment from the nine positive tumor samples (red) and the corresponding sequences from MTCR; MuLVs DG-75, MCF1233, Akv, Moloney, Rauscher and Friend; and a set of representative non-ecotropic proviruses (mERVs). The sequences were aligned using ClustalX, and the corresponding tree was generated using the neighbor-joining method (see Materials and Methods). Bootstrap values (*n* = 1000 trials) are indicated as percentages. Sequences are labeled as xenotropic (X), polytropic (P), modified polytropic (Pm), or ecotropic (E). (B) Phylogenetic tree based on a 2500-nt *pol* PCR fragment from the 9 XMRV-positive tumor samples. The tree was constructed as described in (A).

In addition to the *gag* gene, we also examined the same patient samples for sequence variation in the *pol* gene. We sequenced PCR fragments obtained with a set of primers targeting a 2500-nt stretch in the *pol* gene (Figure S1). Similar to the *gag* fragments, the amplified *pol* fragments were highly similar (Figure 6B) and had >97% nt and >97% aa identity to each other. In contrast, the fragments had <94% nt and <95% aa identity with the most related sequence, that of MuLV DG-75. Interestingly, XMRV-derived *pol* sequences were less similar to and approximately equidistant from the examined representative xenotropic and polytropic endogenous sequences.

Close clustering of the sequenced *gag* and *pol* fragments (Figure 6) indicates that all microarray and RT-PCR positive cases represent infection with the same virus. On the other hand, the degree of sequence variation in the examined fragments is higher than that expected from errors introduced during PCR amplification and sequencing. The frequency of nt misincorporation by Taq polymerase has been estimated as 10^−6^ − 10^−4^ ([63] and references therein), compared with the observed rate of up to 2% in the *gag* and *pol* fragments. These findings suggest that the observed XMRV sequence variation is a result of natural sequence diversity, consistent with the virus being independently acquired by the affected patients, and argue against laboratory contamination as a possible source of XMRV.

RETRACTED

### Detection of XMRV in Tumor-Bearing Prostatic Tissues Using FISH

To localize XMRV within human prostatic tissues, and to measure the frequency of the infected cells, XMRV nucleic acid was visualized using FISH on formalin-fixed prostate tissues. A SpectrumGreen fluorescently labeled FISH probe cocktail spanning all viral genes was prepared using cDNA derived from the XMRV isolate cloned from patient VP35 (Materials and Methods). Distinct FISH-positive cells were observed in the tumors positive for XMRV by RT-PCR (e.g., VP62 and VP88) (Figure 7). To identify cell types associated with the positive FISH signal, the same sections were subsequently stained with hematoxylin and eosin (H&E). Most FISH-positive cells were stromal fibroblasts (Figure 8A), including those undergoing cell division (Figure 8B). In addition, occasional infected hematopoietic cells were also seen (Figure 8C). XMRV FISH with concurrent immunostaining for cytokeratin AE1/AE3 to achieve specific labeling of epithelial cells [64] showed no XMRV-infected cells that also had the epithelium-specific staining, confirming their non-epithelial origin (Figure 8C). While the XMRV nucleic acid was usually present within nuclei (Video S1), suggesting integrated proviral DNA, some cells showed cytoplasmic staining adjacent to the nucleus, suggestive of viral mRNA and/or pre-integration complexes in non-dividing cells (Figure 8A).

**Figure 7:** Detection of XMRV Nucleic Acid in Prostatic Tissues Using FISH Prostatic tumor tissue sections from QQ cases VP62 (A–C) and VP88 (D–F) were analyzed by FISH using DNA probes (green) derived from XMRV VP35 (top right enlargements). Nuclei were counterstained with DAPI. The same sections were then visualized by H&E staining (left panels). Scale bars are 10 μm. Arrows indicate FISH positive cells, and their enlarged images are shown in the bottom right panels.

**Figure 8:** Characterization of XMRV-Infected Prostatic Cells by FISH and FISH/Immunofluorescence Using a tissue microarray, prostatic tumor tissue sections from QQ case VP62 were analyzed by FISH (green) using DNA probes derived from XMRV VP35 (left panels). Nuclei were counterstained with DAPI. The same sections were then visualized by H&E staining (middle panels). Arrows indicate FISH-positive cells, and their enlarged FISH and H&E images are shown in the top right and bottom right panels, respectively. Scale bars are 10 μm. (A) A stromal fibroblast. (B) A dividing stromal cell. (C) A stromal hematopoietic cell. The section was concomitantly stained for XMRV by FISH (green) and cytokeratin AE1/AE3 by immunofluorescence (red).

RETRACTED

We also used FISH to obtain a minimal estimate of the frequency of XMRV-infected prostatic cells. For this purpose we employed a tissue microarray containing duplicates of 14 different prostate cancer tissue specimens (Table 2). FISH with DNA probes derived from XMRV VP35 showed five to ten XMRV/FISH–positive cells (about 1% of prostate cells observed) in each of five homozygous RNase L 462Q (QQ) cases: VP29, 31, 42, 62, and 88. Patient sample VP79, also a QQ case, contained two positive cells (0.4% of total cells examined). All of the XMRV/FISH–positive cells observed were stromal cells. In contrast, three RR tissue samples and two RQ tissue samples showed one or no (<0.15%) FISH-positive cells. Two of the QQ cases, VP35 and VP90, positive by *gag* RT-PCR, showed only one FISH-positive cell each (Table 2). Conversely, one case, VP31, was FISH-positive, but *gag*–RT-PCR negative. As expected, Chromosome 1–specific probes used as a positive control specifically labeled nearly every cell from the examined case VP88, whereas a KSHV-specific probe used as a negative control did not label any cells in sections from cases VP88 and VP51, but did efficiently label 293T cells transfected with KSHV DNA (unpublished data). Thus, consistent with the microarray and RT-PCR data, detection of XMRV by FISH was associated primarily with QQ cases. In addition, in samples where XMRV was detected, all positive cells were stromal and did not account for more than 1% of all prostatic cells. Finally, differences in the numbers of XMRV-positive cells detected in the different samples could be due to heterogeneity in virus copy numbers between different patients and/or specific regions of the prostate sampled.

**Table 2:** Frequency of XMRV-Infected Prostatic Cells Determined by FISH

### Detection of XMRV in Tumor-Bearing Prostatic Tissues Using IHC

To identify cells expressing XMRV proteins, we assayed for the presence of Gag protein using a monoclonal antibody against (SFFV); this antibody is reactive against Gag proteins from a wide range of different ecotropic, polytropic, and xenotropic MuLV strains [65]. Using this antibody, positive signal by IHC was observed in prostatic tissues of XMRV-positive cases VP62 and VP88, both QQ (Figure 9). An enhanced alkaline phosphatase red detection method allowed Gag detection in the same cells with both fluorescence (Figure 9A–9D, left) and bright field (Figure 9A–9D, middle) microscopy. The Gag-expressing cells were observed in prostatic stromal cells with a distribution and frequency similar to that detected by FISH (Figure 9 and unpublished data). In contrast, no Gag-positive cells were observed in VP51 prostatic tissue, which is of RR genotype (Figure 9E).

RETRACTED

**Figure 9:** Detection of XMRV Protein in Prostatic Tissues Using Immunostaining Prostatic tumor tissue sections from QQ cases VP62 (A and B) and VP88 (C and D), as well as an RR case VP51 (E) were stained, then visualized by immunofluorescence (left) or bright field (middle) using a monoclonal antibody to SFFV Gag protein. Nuclei are counterstained with hematoxylin. Enlarged images corresponding to the positive cells are shown on the right. Scale bars are 5 μm in (A), (B), and (E) and 10 μm in (C) and (D).

## Discussion

The results presented here identify XMRV infection in prostate tissue from approximately 40% of patients with prostate cancer who are homozygous for the R462Q variant (QQ) of RNase L, as judged by both hybridization to the Virochip microarray and by RT-PCR with XMRV-specific primers. Parallel RT-PCR studies of prostate tumors from wild-type (RR) and heterozygous (RQ) patients revealed evidence of XMRV in only one of 66 samples, clearly demonstrating that human XMRV infection is strongly linked to decrements in RNase L activity. This result supports the view that the R462Q RNase L variant leads to a subtle defect in innate (IFN-dependent) antiviral immunity.

As its name indicates, XMRV is closely related to xenotropic murine leukemia viruses (MuLVs). Unlike ecotropic MuLVs, such as the canonical Moloney MuLV, which grow only in rodent cells in culture, xenotropic MuLVs can grow in non-rodent cells in culture but not in rodent cell lines. Xenotropic viruses have been isolated from many inbred as well as wild mouse strains. Studies of the distribution of non-ecotropic sequences in different mouse strains show that the diversity of xenotropic proviral sequences in wild mice is greater than that found in the inbred laboratory strains [49,66]. This finding led to the conclusion that these endogenous elements were independently and relatively recently acquired by different mouse species as a result of infection rather than inheritance [49]. Unlike ecotropic MuLVs, which can only recognize a receptor (CAT-1) specific to mouse and rat species [67–69], xenotropic viruses recognize a protein known as XPR1 or SYG1. XPR1 is expressed in all higher vertebrates, including mice, but polymorphisms in the murine gene render it unable to mediate xenotropic MuLV entry [38–40]. Thus, xenotropic MuLVs have a potential to infect a wide variety of mammalian species, including humans.

RETRACTED

Xenotropic MuLVs have occasionally been detected in cultured human cell lines. For example, MuLV DG-75 was cloned from a human B-lymphoblastoid cell line [24], and an infectious xenotropic MuLV was detected in a human small cell lung cancer line NCI-417 [32]. Although laboratory contamination, either in culture or during passage of cell lines in nude mice, cannot be ruled out as a possible source in these cases, such contamination cannot explain our results. The evidence for this is as follows: (i) XMRV was detected in primary human tissues; (ii) no murine sequences (e.g., GAPDH) could be detected in our materials by PCR; (iii) infection was predominantly restricted to human samples with the QQ *RNASEL* genotype; (iv) polymorphisms were found in the XMRV clones recovered from different patients consistent with independent acquisition of the virus by these individuals; and (v) viral nucleic acids and antigens could be detected in infected QQ prostate tissue by FISH and IHC, respectively. Taken together, the above evidence argues strongly against laboratory contamination with virus or cloned DNA material as the source of XMRV infection in the analyzed samples. To our knowledge, this report represents the first published examples of authentic infection of humans with a xenotropic MuLV-like agent. Although our efforts to clone the sites of XMRV integration into the host genome have been limited by the small amounts of prostate tissue available for this purpose, our work to clone such sites is ongoing and will provide an important additional piece of evidence for XMRV infection in humans.

The XMRV sequence is not found in human genomic DNA, and none of the human endogenous retroviruses, including the only known gammaretrovirus-like human endogenous sequences (hERVs E and T) [70], bare any significant similarity to the XMRV genome. This indicates that XMRV must have been acquired exogenously by infection in positive subjects. From what reservoir and by what route such infections were acquired is unknown. It seems unlikely that direct contact with feral mice could explain the observed distribution of infection in our cohort, since there is no reason to believe that rodent exposure would vary according to *RNASEL* genotype. It is possible that infection is more widespread than indicated by the present studies, especially if, as seems likely, individuals with the wild-type RNase L clear infection more promptly than those with the QQ genotype. But if so, a cross-species transfer model of XMRV infection would require improbably high levels of rodent exposure for a developed society like our own. Thus, although the viral sequence suggests that the ultimate reservoir of XMRV is probably the rodent, the proximate source of the infection seems unlikely to be mice or rats. Provisionally, we favor the notion that the XMRV infections we have documented were acquired from other humans, i.e., that XMRV may have been resident in the human population for some time. This speculation will, however, require direct epidemiologic validation. It also remains to be determined if RNase L R462Q homozygotes are more sensitive to the acquisition of infection, or are simply less likely to clear infection once acquired. This is an important issue, since if the latter model is correct, it would imply that in younger humans, XMRV prevalence may be higher than what is observed in our prostate cancer cohort (mean age 58.7 y). We are currently developing serologic assays for use in population-based studies that should shed light on these matters.

RETRACTED

While presented work documents a clear link of XMRV infection to RNase L deficiency, we emphasize that the data we have accumulated does not mandate any etiological link to prostate cancer. Furthermore, our finding that XMRV infection is targeted to stromal cells and not to carcinoma cells and the fact that the XMRV genome harbors no host-derived oncogenes rule out two classical models for retroviral oncogenesis: direct introduction of a dominantly acting oncogene and insertional activation of such a gene. However, more indirect contributions of the virus to the tumor can certainly be envisioned. Recent work has shown that stromal cells have an active role in directly promoting tumorigenesis of adjacent epithelial cells by producing various cytokines and growth factors that serve as proliferative signals [71] or indirectly by modifying the tumor microenvironment by promotion of angiogenesis or recruitment of inflammatory mediators leading to oxidative stress [72]. In particular, cancer-associated fibroblasts stimulate growth of human prostatic epithelial cells and alter their histology in vivo [73]. It is conceivable that XMRV-infected prostatic stromal cells could produce and secrete growth factors, cytokines or other factors that stimulate cell proliferation or promote oxidative stress in surrounding epithelia. Such a paracrine mechanism could still function quite efficiently even with the relatively small number of XMRV-infected cells that characterize the lesion.

RETRACTED

Finally, we note that the identification of an exogenous infection such as XMRV could help explain why not all genetic studies have consistently identified RNase L as a prostate cancer susceptibility factor. If such an infection were linked, however indirectly, to prostate cancer risk, and if the prevalence of infection is not uniform in different populations, populations with low XMRV prevalence might be expected to show no association of *RNASEL* lesions to prostate cancer.

Clearly, resolution of these issues will require much further investigation. We need to determine the prevalence of XMRV infection in the general population, understand its routes of transmission and tissue tropism, explore its associations with pre-maligant and other prostatic conditions, and define the biochemical interactions of the virus with the 2–5A/RNase L system. The availability of molecular clones, infectious virus stocks, and susceptible cell culture systems should greatly enhance our ability to probe these and other questions in the near future.

## Materials and Methods

### Genotyping of patients, and prostate tissue processing.

All human samples used in this study were obtained according to protocols approved by the Cleveland Clinic's Institutional Review Board. Age, clinical parameters, and geographical locations of XMRV-positive prostate cancer cases are provided in Table S3. Men scheduled to undergo prostatectomies at the Cleveland Clinic were genotyped for the R462Q (1385G->A) *RNASEL* variant using a premade TAQMAN genotyping assay (Applied Biosystems, Foster City, California, United States; Assay c_935391_1) on DNA isolated from peripheral blood mononuclear cells. Five nanograms of genomic DNA were assayed according to the manufacturer's instructions, and analyzed on an Applied Biosystems 7900HT Sequence Detection System instrument. Immediately after prostatectomies, tissue cores were taken from both the transitional zone (the site of benign prostatic hyperplasia, BPH) and the peripheral zone (where cancer generally occurs), snap-frozen in liquid nitrogen, and then stored at −80 °C. Remaining prostate tissue was fixed in 10% neutral buffered formalin, processed, and embedded in paraffin for later histological analyses. Frozen tissue cores were transferred from dry ice immediately to TRIZOL reagent (Invitrogen, Carlsbad, California, United States), homogenized with a power homogenizer or manually using a scalpel followed by a syringe, and total RNA was isolated according to the manufacturer's instructions. The prostate tissue RNA was then subjected to RNase-free DNase I (Ambion, Austin, Texas, United States) digestion for 30 min at 37 °C. The sample was then extracted with phenol and the RNA was precipitated with isopropanol overnight at −20 °C followed by centrifugation at 12,000 g for 30 min at 4 °C. Poly-A RNA was isolated from the DNase digested total RNA using the Oligotex mRNA Midi Kit (Qiagen USA, Valencia, California, United States) as instructed by the manufacturer. The poly-A RNA concentration was measured using the RIBOgreen quantitation kit (Molecular Probes, Invitrogen), and the samples were stored at −80 °C**.**

RETRACTED

### Microarray screening.

Virochip microarrays used in this study were identical to those previously described [20–22]. Prostate tumor RNA samples were amplified and labeled using a modified Round A/B random PCR method and hybridized to the Virochip microarrays as reported previously (Protocol S1 in [21]). Microarrays were scanned with an Axon 4000B scanner (Axon Instruments, Union City, California, United States) and gridded using the bundled GenePix 3.0 software. Microarray data have been submitted to the NCBI GEO database (GSE3607). Hybridization patterns were interpreted using E-Predict as previously described [22] (Table S1). To make Figure 1, background-subtracted hybridization intensities of all retroviral oligonucleotides (205) were used to cluster samples and the oligonucleotides. Average linkage hierarchical clustering with Pearson correlation as the similarity metric was carried out using Cluster (version 2.0) [74]. Cluster images were generated using Java TreeView (version 1.0.8) [75].

### Genome cloning and sequencing.

Amplified and labeled cDNA from the VP35 tumor sample was hybridized to a hand-spotted microarray containing several retroviral oligonucleotides, which had high hybridization intensity on the Virochip during the initial microarray screening. Nucleic acid hybridizing to two of the oligonucleotides (9628654_317_rc derived from MTCR: TTC GCT TTA TCT GAG TAC CAT CTG TTC TTG GCC CTG AGC CGG GGC CCA GGT GCT CGA CCA CAG ATA TCC T; and 9626955_16_rc derived from SFFV: TCG GAT GCA ATC AGC AAG AGG CTT TAT TGG GAA CAC GGG TAC CCG GGC GAC TCA GTC TGT CGG AGG ACT G) was then individually eluted off the surface of the spots and amplified by PCR with Round B primers. Preparation of the hand-spotted array, hybridization, probe recovery, and PCR amplification of the recovered material were carried out according to Protocol S1. The recovered amplified DNA samples were then cloned into pCR2.1-TOPO TA vector (Invitrogen), and the resulting libraries were screened by colony hybridization with the corresponding above oligonucleotides as probes. Hybridizations were carried out using Rapid-Hyb buffer (Amersham, Piscataway, New Jersey, United States) according to the manufacturer's protocol at 50 °C for 4 h. Eight positive clones were sequenced, of which two (one from each library; clones K1 and K2R1 in Figure 2A) were viral and had 94–95% nt identity to MTCR.

RETRACTED

To sequence the remainder of the VP35 genome as well as the entire genome from the VP42 tumor, we amplified fragments of the genome by PCR using either amplified (Round B) or unamplified (Round A) cDNA prepared for original Virochip screening. This was accomplished first using a combination of primers derived from the sequence of MTCR and earlier recovered clones of XMRV. The two overlapping fragments from VP62 were amplified by PCR from cDNA generated by priming poly-A RNA with random hexamers. All PCR primers are listed in Table S2. The amplified fragments were cloned into pCR2.1-TOPO TA vector (Invitrogen) and sequenced using M13 sequencing primers. Genome assembly was carried out using CONSED version 13.84 for Linux [76].

### PCR.

Screening of tumor samples by *gag* nested RT-PCR was carried out according to Protocol S2. PCR fragments in all positive cases were gel-purified using QIAEX II gel extraction kit (Qiagen), cloned into pCR2.1-TOPO TA vector (Invitrogen), and sequenced using M13 sequencing primers.

*Pol* PCR was carried out using amplified cDNA (Round B material) as the template.

Sequence of the primers used for amplification (2670F, 3870R, 3810F, and 5190R) is listed in Table S2. Amplified products were gel-purified using QIAEX II gel extraction kit (Qiagen), and purified products were directly used for sequencing.

### Phylogenetic analyses.

Xenotropic mERV Chromosome 1, xenotropic mERV Chromosome 4, and xenotropic mERV Chromosome 9 were chosen by BLAST querying the NCBI nr database with the complete XMRV genomes and selecting the most similar full-length proviral sequences, all of which happened to have xenotropic envelopes (Figure S2C). Polytropic mERV Chromosome 7 and polytropic mERV Chromosome 11 were chosen by selecting NCBI nr full-length proviral sequences with envelopes most similar to a prototype polytropic clone MX27 [77]. Similarly, modified polytropic mERV Chromosome 7 and modified polytropic mERV Chromosome 12 were selected on the basis of similarity to a prototype-modified polytropic clone MX33 [77]. U3 analysis was performed using previously described reference sequences: Mcv18, Mcv3, Mxv2, Mcv11, Mxv11, and HEMV18 [49]; CWM-T-15, CWM-T-15–4, CWM-T-25a, and CWM-T-25b [48].

To generate the neighbor-joining tree of complete genomic sequences (Figure 3), the sequences were first manually edited to make all genomes the same length, i.e., R to R. The edited sequences were then aligned with ClustalX version 1.82 for Linux [78,79] using default settings. The tree was generated based on positions without gaps only; Kimura correction for multiple base substitutions [80] and bootstrapping with *n* = 1000 were also used.

RETRACTED

All other trees were generated as above, except sequences were first trimmed to the same length, gaps were included, and Kimura correction was not used, as using these parameters did not have any significant effect on the trees.

### Antibodies.

Monoclonal antibody to SFFV Gag protein was produced from R187 cells ([65]; ATCC: CRL-1912) grown in DMEM (Media Core, Cleveland Clinic Foundation, Cleveland, Ohio, United States) with 10% ultra-low IgG FBS (Invitrogen) until confluent. Conditioned media was collected every three days from confluent cultures. Five ml of conditioned media per preparation was centrifuged at 168 × g for 5 min at 4 °C. Supernatant was filtered through a 0.22-μm syringe filter unit (Millipore, Billerica, Massachusetts, United States) and concentrated 16-fold in an Amicon ultrafiltration unit with a 100-kDa molecular weight cutoff membrane (Millipore). Sodium azide was added to a final concentration of 0.02%. Concomitant XMRV FISH/cytokeratin immunofluorescence was performed using a mouse anti-cytokeratin AE1/AE3 (20:1 mixture) monoclonal antibody (Chemicon International, Temecula, California, United States) capable of recognizing normal and neoplastic cells of epithelial origin.

### FISH.

The XMRV-35 FISH probe cocktail was generated using both 2.15-kb and 1.84-kb segments of the viral genome obtained by PCR with forward primer-2345, 5′ ACC CCT AAG TGA CAA GTC TG 3′ with reverse primer-4495, 5′ CTG GAC AGT GAA TTA TAC TA 3′ and forward primer-4915, 5′ AAA TTG GGG CAG GGG TGC GA 3′ with reverse primer-6755, 5′ TTG GAG TAA GTA CCT AGG AC 3′, both cloned into pGEM-T (Promega, Madison, Wisconsin, United States). The recombinant vectors were digested with *EcoR*I to release the viral cDNA fragments, which were purified after gel electrophoresis (Qiagen). The purified viral cDNA inserts were used in nick translation reactions to produce SpectrumGreen dUTP fluorescently labeled probe according to manufacturer's instructions (Vysis Inc., Des Plaines, Illinois, United States). Freshly baked slides of prostatic tissues or tissue microarray arrays with ~4-μm thick tissue sections were deparaffinized, rehydrated, and subjected to Target Retrieval (Dako, Glostrup, Denmark) for 40 min at 95 °C. Slides were cooled to room temperature and rinsed in H_2_O. Proteinase K (Dako) at 1:5000 in Tris-HCl (pH 7.4) was applied directly to slides for 10 min at room temperature. Adjacent tissue sections were also probed with SpectrumGreen dUTP fluorescently labeled KSHV-8 DNA (nts 85820–92789) as a negative control or, as a positive control with SpectrumGreen and SpectrumOrange labeled TelVysion DNA Probe cocktail (Vysis), specific for subtelomeric regions of the P and Q arms of human Chromosome 1 as a positive control to ensure the tissue was completely accessible to FISH. FISH slides were examined using a Leica DMR microscope (Leica Micro-Systems, Heidelberg, Germany), equipped with a Retiga EX CCD camera (Q-Imaging,Vancouver, British Columbia, Canada). FISH images were captured using a Leica TCS SP2 laser scanning confocal with a 63× oil objective numerical aperature 1.4 (Leica Micro-Systems) microscope. XMRV nucleic acids were visualized using maximum intensity projections of optical slices acquired using a 488-nm argon-laser (emission at 500–550 nm). TelVysion DNA Probes were visualized using maximum intensity projections of optical slices acquired using a 488-nm argonlaser (emission at 500–550 nm) and 568-nm krypton-argon-laser (emission at 575–680 nm). DAPI was visualized using maximum intensity projections of optical slices acquired using a 364–nm UV-laser (emission at 400–500 nm). Slides were subsequently washed in 2× SSC (0.3 M sodium chloride and 0.03 M sodium citrate, [pH 7.0]) to remove coverslips, and H&E stained for morphological evaluation.

RETRACTED

### IHC.

IHC on human tissues was performed on a Benchmark Ventana Autostainer (Ventana Medical Systems, Tucson, Arizona, United States). Unstained, formalin-fixed, paraffin-embedded prostate sections were placed on electrostatically charged slides and deparaffinized followed by a mild cell conditioning achieved through the use of Cell Conditioner #2 (Ventana Medical Systems). The concentrated R187 monoclonal antibody against SFFV p30 Gag was dispensed manually onto the sections at 10 μg per ml and allowed to incubate for 32 min at 37 °C. Endogenous biotin was blocked in sections using the Endogenous Biotin Blocking Kit (Ventana Medical Systems). Sections were washed, and biotinylated ImmunoPure Goat Anti-Rat IgG (Pierce Biotechnology, Rockford, Illinois, United States) was applied at a concentration of 4.8 μg per ml for 8 min. To detect Gag protein localization, the Ventana Enhanced Alkaline Phosphatase Red Detection Kit (Ventana Medical Systems) was used. Sections were briefly washed in distilled water and counterstained with Hematoxylin II (Ventana Medical Systems) for approximately 6 min. Sections were washed, dehydrated in graded alcohols, incubated in xylene for 5 min, and coverslips were added with Cytoseal (Microm International, Walldorf, Germany). Negative controls were performed as above except without the addition of the R187 monoclonal antibody.

RETRACTED

Concomitant XMRV FISH/cytokeratin IHC was performed on slides of prostate tissue from patient VP62. First, sections were immunostained for cytokeratin AE1/AE3 using the Alexa Fluor 594 Tyramide Signal Amplification Kit (Molecular Probes, Invitrogen). Briefly, unstained, formalin-fixed, paraffin-embedded sections cut at ~4 μm were placed on electrostatically charged slides, baked at 65 °C for at least 4 h, deparaffinized in xylene, and rehydrated through decreasing alcohol concentrations. Slides were incubated in Protease II (Ventana Medical Systems) for 3 min at room temperature and washed in phosphate-buffered saline (PBS) in peroxidase quenching buffer (PBS + 3% H_2_O_2_) for 60 min at room temperature, then incubated with 1% blocking reagent (10 mg/ml BSA in PBS) for 60 min at room temperature. The slides were incubated with cytokeratin AE1/AE3 antibody diluted in 1% blocking reagent for 60 min at room temperature and rinsed 3× times in PBS. Goat anti-mouse IgG-horseradish peroxidase (Molecular Probes, Invitrogen) was added and incubated for 60 min at room temperature. The slides were rinsed 3× in PBS. The tyramide solution was added to the slides for 10 min at room temperature and the slides were rinsed 3× in PBS. Slides were then placed in Target Retrieval solution (Dako) for 40 min at 95 °C. FISH for XMRV was performed as described above except in the absence of proteinase K treatment. After FISH, the slides were mounted with Vectashield Mounting Medium plus DAPI (Vector Labs, Burlingame, California, United States) and examined using fluorescence microscopy. Immunofluorescence images were captured using a Texas red filter with a Leica DMR microscope (Leica Micro-Systems), equipped with a Retiga EX CCD camera (QImaging).

## Supporting Information

Figure S1 Complete Nucleotide Sequence of XMRV VP35 Numbers to the left indicate nt coordinates relative to the first nt. Predicted open reading frames for Gag, Gag-Pro-Pol, and Env polyproteins are shown below the corresponding nt. Characteristic 24-nt deletion in the 5′ *gag* leader is indicated with a triangle. Other genome features as well as primers used in the nested *gag* RT-PCR are shown as arrows.
(558 KB PDF)

Figure S2 Phylogenetic Analysis of XMRV Based on Predicted Gag, Pro-Pol, and Env Polyproteins Predicted Gag (A), Pro-Pol (B), and Env (C) sequences of XMRV VP35, VP42, and VP62 (red) as well as the corresponding sequences from MTCR; MuLVs DG-75, MCF1233, Akv, Moloney, Friend, and Rauscher; feline leukemia virus (FLV); koala retrovirus (KoRV); gibbon ape leukemia virus (GALV), and a set of representative non-ecotropic proviruses (mERVs) were aligned using ClustalX. The resulting alignments were used to generate unrooted neighbor-joining trees (see Materials and Methods). Sequences are labeled as xenotropic (X), polytropic (P), modified polytropic (Pm), or ecotropic (E).
(186 KB EPS)

Figure S3 Comparison of XMRV U3 Region to Representative Non-Ecotropic Sequences (A) Multiple sequence alignment of U3 sequences from XMRV VP35, VP42, and VP62; MuLVs NZB-9–1 and NFS-Th-1; and from representative non-ecotropic proviruses [37,48,49]. The sequences were aligned using ClustalX (see Materials and Methods). Only sequences most similar to XMRV are shown. Glucocorticoid response element (GRE), and TATA and CAT boxes are indicated by lines. Direct repeat regions (boxed) are numbered according to the existing convention [37,49]. Triangle indicates a 190 nt insertion in polytropic proviruses [37]. XMRV-specific AG dinucleotide insertion is shown in red. Dots denote nt identical to those from XMRV, and deleted nt appear as spaces.
(B) Phylogenetic tree based on U3 nt sequences. Multiple sequence alignment from (A) was used to generate an unrooted neighbor-joining tree (see Materials and Methods). Bootstrap values (*n* = 1000 trials) are shown as percentages. U3 sequences from XMRV are shown in red.
(188 KB EPS)

Protocol S1 Probe Recovery from Hand-Spotted Microarrays by “Scratching” (83 KB PDF)

Protocol S2 XMRV *gag* Nested RT-PCR (172 KB PDF)

Table S1 Computational Viral Species Predictions Using E-Predict for the Virochip Microarrays Shown in Figure 1
(48 KB DOC)

Table S2 PCR Primers Used for Sequencing of XMRV Genomes (45 KB DOC)

Table S3 Age, Clinical Parameters, and Geographical Locations of XMRV-Positive Prostate Cancer Cases (39 KB DOC)

Video S1 Confocal Optical Image Planes of a Representative XMRV FISH Positive Cell Optical image planes (0.5 μm step-size) of the XMRV FISH positive cell from Figure 1A acquired using a Leica TCS SP2 laser scanning spectral confocal microscope (Leica, Heidelberg, Germany) were reconstructed into a 3D volume set using Volocity 3.5 (Improvision, Lexington, Massachusetts, United States). Using Volocity's movie sequence editor, each volume was rotated along horizontal and vertical axes, adjusting nuclei stained DAPI (blue) channel brightness to visualize underlying XMRV FISH (green) nucleic acid signal. The resulting image frames were exported as a movie sequence. Underlying grid represents glass slide to which tissue was placed for FISH analysis. Each square unit within grid represents 4 μm in height and width.
(237 KB WMV)

RETRACTED

### Accession Numbers

Accession numbers from Gen Bank (http://www.ncbi.nlm.nih.gov/Genbank) are: AKV MuLV (J01998), feline leukemia virus (NC_001940), Friend MuLV (NC_001372), gibbon ape leukemia virus (NC_001885), koala retrovirus (AF151794), modified polytropic mERV Chromosome 7 (AC127565; nt 64,355–72,720), modified polytropic mERV Chromosome 12 (AC153658; nt 85,452–93,817), Moloney MuLV (NC_001501), MTCR (NC_001702MuLV DG-75 (AF221065); MuLV MCF 1233 (U13766), MuLV NCI-417 (AAC97875), MuLV NZB-9–1 (K02730), polytropic mERV Chromosome 7 (AC167978; nt 57,453–65,805), polytropic mERV Chromosome 11 (168–229,176,580), prototype polytropic clone MX27 (M17327), Rauscher MuLV (NC_001819), xenotropic mERV Chromosome 1 (AC083892, nt 158,240–166,448), xenotropic mERV Chromosome 4 (AL627077; nt 146,400–154,635), xenotropic mERV Chromosome 9 (AC121813; nt 37,520–45,770), XMRV VP35 (DQ241301), XMRV VP42 (DQ241302), and XMRV VP 62 (DQ399707). 

## Abbreviations

2–5A: 5′-phosphorylated 2′-5′ oligoadenylate
aa: amino acid
FISH: fluorescence in situ hybridization
H&E: hematoxylin and eosin
HPC: hereditary prostate cancer
IFN: interferon
IHC: immunohistochemistry
LTR: long terminal repeat
MCF: mink cell focus-inducing murine leukemia virus
MTCR: murine type C retrovirus
MuLV: murine leukemia virus
nt: nucleotide(s)
NZB-9–1: New Zealand Black 9–1 xenotropic retrovirus
ORF: open reading frame
PBS: phosphate-buffered saline
PCR: polymerase chain reaction
QQ: *RNASEL* homozygous R462Q
QR: *RNASEL* heterozygous R462Q
RNase L: Ribonuclease L
RR: *RNASEL* homozygous wild-type
SFFV: spleen focus-forming virus
VR: variable region
XMRV: xenotropic MuLV-related virus
XPR1: xenotropic and polytropic retrovirus receptor
